The article "Head and Neck Squamous Cell Carcinoma: NT5E Could Be a Prognostic Biomarker" was published in 2022. Journal: Appl Bionics Biomech.

# Head and Neck Squamous Cell Carcinoma: NT5E Could Be a Prognostic Biomarker

**DOI:** 10.1155/2022/3051907

**Published:** 2022-04-25

**Authors:** Yaoting Zhang, Sultan Kadasah, Jiaheng Xie, Dongsheng Gu

**Affiliations:** ^1^Department of Otorhinolaryngology-Head and Neck Surgery, The Affiliated Huaian No.1 People's Hospital of Nanjing Medical University, Huaian, 223300 Jiangsu, China; ^2^Department of Biology, Faculty of Science University of Bisha, Bisha, Saudi Arabia; ^3^Department of Burn and Plastic Surgery, The First Affiliated Hospital of Nanjing Medical University, Nanjing, Jiangsu, China

## Abstract

Head and neck squamous cell carcinoma (HNSCC) is a type of tumour with a relatively poor prognosis. In recent years, immune checkpoint inhibitors, such as CTLA-4 and PD-1/PDL-1 inhibitors, have improved the treatment status of advanced tumours. However, the emergence of drug resistance has brought difficulties to clinical treatment, and new immune checkpoint research is imminent. The hypoxia-adenosine pathway, in which CD73 encoded by the NT5E gene is a key enzyme for adenosine production, has been identified as an immune checkpoint of great potential. Therefore, NT5E may play an important role in HNSCC. We performed a detailed bioinformatics analysis of NT5E in HNSCC, and the results showed that the overexpression of NT5E in HNSCC was associated with poor prognosis. Our further investigation of the coexpression pattern of HNSCC could provide a reference for drug resistance and immunotherapy studies.

## 1. Introduction

Adenosine is produced by removing a phosphoric acid molecule from AMP and is involved in numerous critical biological processes in the human body, such as substance metabolism, inflammation regulation, and tumour immunity [1–3]. By acting on different adenosine receptors, adenosine can activate the G-protein coupled receptor pathway, the PI3K/Akt/mTOR pathway, and the MAPK pathway [4]. The key enzyme for the hydrolysis of AMP in the synthesis of adenosine is CD73, which is encoded by NT5E. CD73 is also known as ecto-5′-nucleotidase [5]. Structurally, CD73 is a homodimer linked by disulfide bonds and has a glycosylated N-terminal [6]. It can be anchored to cell membranes by phosphatidylinositol or dissolved in various body fluids [7]. Because of the extensive prospect of the adenosine signalling pathway in oncology research, NT5E is considered a new target for cancer therapy in the future [8].

Head and neck squamous cell carcinoma (HNSCC) is a type of tumour originating in the oral, oropharyngeal, nasopharyngeal, larynx, and hypopharyngeal squamous epithelium, which has a relatively poor prognosis [9]. Recurrent oral ulcers, foreign body sensation, dysphonia, swallowing pain, nasal congestion, nosebleeds, hoarseness, and restricted movement are common clinical manifestations of HNSCC. HNSCC became the seventh most common tumour worldwide in 2018, with 890,000 new cases and 450,000 deaths that year [10]. HPV infection is associated with a part of the HNSCC patients, depending on the cause of the disease, HNSCC can be divided into HPV-positive HNSCC and HPV-negative HNSCC [11]. HPV-positive HNSCCs have a better prognosis than HPV-negative tumours. The five-year survival rate for patients with advanced HPV-positive HNSCC was 75–80%, compared with less than 50% for patients with HPV-negative HNSCC in the same stage. This is because different HPV infection states show different sensitivity to chemotherapy, radiation therapy, and immunotherapy. Some clinical trials have shown that HPV-positive HNSCC patients respond better to chemotherapy, radiation, and immunotherapy than HPV-negative patients. Currently, the efficacy of conventional treatment regimens for HNSCC is not satisfactory, and in this context, the exploration of immunotherapy is gaining momentum [12, 13]. Therefore, it is of great value to find an effective index and explore its significance in HNSCC. The important role of NT5E in many cancers has been demonstrated. However, the study of NT5E in HNSCC is insufficient.

In this study, we first investigated the expression of NT5E (the gene encoding CD73) in HNSCC by database mining. Subsequently, we investigated the correlation between NT5E and HNSCC in terms of clinical characteristics, prognosis, coexpression pattern, and immune infiltration. Thus, our study can provide a new idea for the treatment and drug resistance management of HNSCC.

## 2. Methods

### 2.1. UALCAN

UALCAN (http://ualcan.path.uab.edu) is an open, easy-to-use web tool that provides a convenient platform for exploring TCGA and CPTAC databases [14]. With UALCAN, users can perform comprehensive gene analysis, such as expression profile analysis, clinical characteristics analysis, survival analysis, and pan-cancer analysis. We used the “TCGA Analysis” function of UALCAN to analyse the expression profile of NT5E in various cancers, the correlation of the clinical features of NT5E in HNSCC, the prognostic correlation between NT5E and HNSCC, and the coexpression pattern of NT5E in HNSCC.

### 2.2. GEPIA 2.0

Gene Expression Profiling Interactive Analysis Version 2.0 (GEPIA 2.0, http://gepia2.cancer-pku.cn) is a publicly accessible web-based analysis tool that incorporates high-throughput sequencing data from the TCGA and GTEX databases [15]. We used the “Expression Analysis” function of GEPIA 2.0 to analyse the expression of NT5E in various cancers, the expression of NT5E in HNSCC, and the relationship between NT5E and HNSCC prognosis.

### 2.3. Oncomine

DNA microarray technology has greatly promoted the development of genomics. Oncomine (http://www.oncomine.org/s) is an online database of DNA microarray data [16]. To increase the credibility of the results, we used Oncomine to verify the expression results analysed by UALCAN and GEPIA 2.0.

### 2.4. R Software

R software is a powerful data analysis software. We used R software to process the data of the HNSCC and the normal group from TCGA. In addition, the software package “Clusterprofiler” was used for Gene Ontology (GO) and Kyoto Encyclopedia of Genes and Genomes (KEGG) enrichment analyses of the coexpressed genes.

### 2.5. STRING and Cytoscape Software

The STRING database (https://string-db.org/) is an online search database for known protein interactions [17]. We analysed the protein interactions of coexpressed genes using the STRING database and visualised them using Cytoscape.

### 2.6. TIMER

Tumour immune estimation resource (TIMER) is a web tool that uses deconvolution methods to calculate immune correlation in tumours [18]. We used TIMER to explore the association of NT5E with individual immune cells in HNSCC, HPV-positive HNSCC, and HPV-negative HNSCC.

## 3. Results

### 3.1. Expression of NT5E across Cancers

First, Figure 1(a) obtained in UALCAN showed that NT5E is highly expressed in various cancers, including HNSCC (*P* < 0.05). Then, the “Expression Profile Analysis” in GEPIA 2.0 also showed that NT5E was significantly expressed in HNSCC (Figure 1(b), *P* < 0.05). Finally, the “gene overview” in Oncomine proved the same result (Figure 1(c), *P* < 0.05). Hence, the results of the three databases showed that NT5E was highly expressed in HNSCC compared with normal tissues, and the difference was statistically significant (*P* < 0.05). Therefore, NT5E deserves further exploration in HNSCC.

### 3.2. Relationship between NT5E Expression and Patient Status of HNSCC

Figure 2(a) shows a high expression of NT5E in HNSCC obtained from the GEPIA “Box plots” module, and Figure 2(b) (from UALCAN) exhibits the same result. We then investigated whether NT5E expression was associated with HPV infection status or TP53 mutation status, and the results showed that NT5E expression was more significant in HPV-negative HNSCC (Figure 2(c), *P* < 0.05) and TP53-mutant HNSCC (Figure 2(d), *P* < 0.05). We also explored the relationship between NT5E and methylation level, and the results showed that compared with normal tissues, NT5E had a higher degree of methylation in HNSCC (Figure 2(e), *P* < 0.05), which was more reflected in TP53 nonmutant HNSCC (Figure 2(f), *P* < 0.05).

### 3.3. Survival Analysis of NT5E

Survival analysis of NT5E was performed by two methods (GEPIA 2.0 and UALCAN) to reduce bias. First, the GEPIA analysis (Figure 3(a)) revealed that increased NT5E expression was associated with a worse overall survival rate in patients with HNSCC (*P* = 0.004). However, high expression of NT5E had no significant effect on HNSCC disease-free survival (*P* = 0.11, Figure 3(b)). Then, we plotted a K-M curve using UALCAN (Figure 3(c)), showing that NT5E was associated with poor prognosis in HNSCC (*P* = 0.022). Therefore, NT5E is a potent prognostic marker for HNSCC.

### 3.4. Analysis of NT5E Coexpression Pattern

The “Correlation” function in UALCAN can analyse the coexpressed genes of NT5E and display the top 100 related genes as heat maps (Figures 3(d)–3(g)). These genes were sequenced based on the correlation coefficient. Figures 3(d)–3(g) depict the top 25 genes, the top 26–50 genes, the top 51–75 genes, and the top 76–100 genes, respectively. These 100 genes constituted the coexpression pattern of NT5E. Studying the function of these 100 genes will deepen our understanding of the role of NT5E in HNSCC.

### 3.5. Gene Ontology (GO) and Kyoto Encyclopedia of Genes and Genomes (KEGG) Enrichment Analyses of Genes Coexpressed with NT5E

GO enrichment analysis (Figure 4(a)) can be divided into three subgroups: biological process (BP), cellular component (CC), and molecular function (MF). First, in BP, we find that those coexpressed genes were enriched in cell-substrate adhesion, extracellular matrix organisation, extracellular structure organisation, cell junction assembly, and ameboid-type cell migration. The coexpressed genes were then enriched in the cell-substrate junction, focal adhesion, and collagen-containing extracellular matrix in the CC. Finally, cadherin-binding, actin-binding, actin filament binding, and other genes were enriched in coexpressed genes in MF.

KEGG enrichment analysis (Figure 4(b)) showed that coexpressed genes were mainly concentrated in focal adhesion, PI3K-Akt signalling pathway, regulation of actin cytoskeleton, proteoglycans in cancer, ECM-receptor interaction, MAPK signalling pathway, small cell lung cancer, and bacterial invasion of epithelial cells.

### 3.6. Protein-Protein Interaction Network

Using STRING, we constructed a protein*-*protein interaction network of genes coexpressed with NT5E and visualised it, using Cytoscape. From this network, we can see the interaction in the coexpression mode of NT5E. The more lines that connect, the more interactions occur, which means the gene may be more important. Besides, using the “CytoHubba” plug-in, we screened out 20 hub genes according to the MCC score, as shown in Figure 4(c).

### 3.7. Correlation Analysis of NT5E and Immune Cells in HNSCC

Many genes play essential roles in the immune microenvironment of tumours, and these genes may be targets for future immunotherapy. At the same time, different immune responses due to HPV infection status are the underlying reasons for the difference in the prognosis of HNSCC. To investigate the role of NT5E in the immune microenvironment of HNSCC, we used a data algorithm to calculate the correlation between NT5E and immune cell infiltration. Firstly, we used TIMER to study the immune correlation of NT5E in the whole HNSCC, and the results (Figure 5(a)) showed that the expression of NT5E was significantly correlated with B cells, CD8^+^ T cells, CD4^+^ T cells, neutrophils, and dendritic cells. However, different HPV infection statuses can affect immune function, so it is necessary to analyse HPV-positive HNSCC and HPV-negative HNSCC separately. The results showed that the NT5E expression was more strongly associated with immune infiltration in HPV-negative HNSCC (Figure 5(c)) than in HPV-positive HNSCC (Figure 5(b)).

### 3.8. Validation of NT5E Expression in an Independent Cohort

To further verify the accuracy of our results, we validated the expression of NT5E in an independent cohort. We used the “Ginos Head-Neck” cohort in the Oncomine database to analyse, which is independent of the TCGA cohort. The results showed that NT5E was highly expressed in HNSCC compared with normal tissues (*P* = 5.03E − 7, Figure 6).

## 4. Discussion

In recent years, the advance of immunotherapy has undoubtedly brought hope for refractory tumours. Immune checkpoint inhibitors, such as CTLA-4 and PD1/PDL1 inhibitors, have demonstrated clinical efficacy in many tumours, which is a major breakthrough in oncology [19]. However, there are still many patients who are not sensitive to the existing immune checkpoint inhibitors, so it is necessary to explore new immune checkpoints [20]. The hypoxia-adenosine pathway is considered one of the most promising new immune checkpoint pathways [21]. In this pathway, CD73 protein encoded by NT5E is the crucial enzyme for the hydrolysis of AMP to adenosine [5]. As a result, NT5E has been identified as a potential therapeutic target. Hence, we selected the NT5E gene, which encodes CD73, as the study object to explore its potential role in HNSCC.

In this study, first, we found that NT5E is highly expressed in many cancers, including HNSCC. Second, we discovered that NT5E was more closely related to HPV-negative HNSCC and TP53-mutated HNSCC. Further analysis revealed that NT5E had a higher level of methylation in the HNSCC compared to normal tissue. Moreover, survival analysis found that high expression of NT5E can decrease the overall survival in patients with HNSCC. Hence, high expression of NT5E could also be used as a poor prognostic indicator for HNSCC. In the analysis of the coexpression pattern of NT5E, coexpressed genes mainly accumulate in the extracellular matrix organisation, focal adhesion, PI3K-Akt signalling pathway, MAPK signalling pathway, and others. This suggests that NT5E may have other potential functions. In addition, we found 20 hub genes in the protein interaction network, including ITGA6, ITGA3, ITGA5, ITGB1, ITGB4, LAMA3, LAMB3, LAMC, PXN, and CD44, which provided new directions for further exploring the function of NT5E.

Tumours that are difficult to treat tend to lack a valid prognostic marker. Significant biomarkers often play an important role in the genesis and progression of tumours. Therefore, finding a valuable indicator and studying the relevant treatment plan can improve the clinical effect and survival rate. NT5E is a valuable biomarker for HNSCC, and its high expression is associated with a poor prognosis of HNSCC.

HPV-negative patients, who often have a long history of alcohol abuse and smoking, tend to have a poor prognosis [22]. On the contrary, patients with HPV-positive HNSCC, whose pathogenic mechanism is viral gene insertion, tend to have a better prognosis [23]. Immunosuppression and refractory drug resistance are more likely to occur in patients who are HPV-negative [24]. NT5E was more significantly expressed in HPV-negative HNSCCs, undoubtedly providing a potential new therapeutic direction for this patient subgroup.

Although CD73 has long been considered an AMPase, it has recently been found that CD73 has more than that catalysis function [25]. CD73 has been proposed to be related to the adhesion of the extracellular matrix (ECM), mediating the migration and metastasis of tumour cells, and also involved in the epithelial-mesenchymal transformation (EMT) of tumours [26–28]. Our study also found that the coexpression mode of NT5E is enriched in cell-substrate adhesion, extracellular matrix organisation, extracellular structure organisation, cell junction assembly, and ameboid-type cell migration. This undoubtedly reveals the role of CD73 in the tumour microenvironment. ECM is an important molecule in the tumour microenvironment. Cell-ECM adhesion can not only increase tumour invasion ability but also activate a series of signalling pathways [29].

Drug resistance in HNSCC has always been a challenging problem in oncology therapy [30]. Many studies have proved focal adhesion to be one of the important mechanisms of tumour resistance development [31]. KEGG enrichment analysis of NT5E coexpressed genes showed a correlation with focal adhesion, suggesting that NT5E may be involved in the formation of drug resistance in HNSCC, which provides a reference for future treatment studies. Similarly, overactivation of the PI3K-Akt pathway is also an important mechanism of tumour growth and invasion, which shows the role of NT5E in tumour progression and suggests that NT5E is a potential target [32–34]. In general, NT5E is associated with immunosuppression of tumours [5], but we used TIMER analysis to show that NT5E is more strongly related to infiltration of many immune cells in HPV-negative HNSCCs, which have a poorer prognosis compared with HPV-positive HNSCC. This could lead to novel approaches to HNSCC immunotherapy in the future.

At present, many studies have preliminarily elucidated the role of CD73 in cancer. Ma et al. found that CD73 maintains tumour stem cell characterization of hepatocellular carcinoma by upregulating SOX9 expression [35]. Chen et al. found that CD73 is a novel prognostic marker of pancreatic cancer and is associated with immune escape [36]. Kim et al. found that CD73 may be a novel immunotherapy target for colorectal cancer [37]. Therefore, CD73 is of great value in future cancer treatment.

All in all, our study could provide a meaningful biomarker for HNSCC. However, there are limitations to our study. First, we lack in-depth experiments to verify the results of the paper. Additionally, using multiple databases increases the reliability of the results besides increasing the background heterogeneity. We will correct these problems in future research.

## 5. Conclusion

For tumours such as HNSCC with a relatively poor prognosis, it is critical to find an excellent biomarker. In our study, NT5E was found to be overexpressed in HNSCC and was associated with a poor prognosis. Furthermore, we found that the coexpression pattern of NT5E is related to cell-ECM adhesion and focal adhesion, which may provide a reference for drug resistance research. In the future, it is hoped that more high-quality studies will elucidate the powerful role of CD73, the protein encoded by NT5E.

## Figures and Tables

**Figure 1:** (a) Expression of NT5E across TCGA cancers. The results showed that NT5E was highly expressed in HNSCC compared with normal tissues (*P* < 0.05). (b) Differential expression of NT5E in multiple cancers in GEPIA database. The red tumor type represents the upregulated expression of NT5E, the green tumor type represents the downregulated expression of NT5E, and the black tumor type represents the difference of no statistical significance. We can see that NT5E is upregulated in HNSCC. (c) Overview of NT5E in multiple cancers in Oncomine database. Red represents upregulation, blue represents downregulation, and the numbers in the figure represent “fold change.” We can see that NT5E expression is upregulated in HNSCC, with fold change of 3.

**Figure 2:** (a) Expression of NT5E in HNSC is significantly higher than normal tissues (GEPIA): analysis of 519 HNSCCs and 44 normal tissues showed that NT5E was significantly overexpressed in HNSCC (*P* < 0.05). (b) Expression of NT5E in HNSC based on sample types (UALCAN) showed that NT5E was significantly overexpressed in HNSCC (*P* < 0.05). (c) Expression of NT5E in HNSC based on HPV status: NT5E expression was more significant in HPV-negative HNSCC (*P* < 0.05) (d) Expression of NT5E in HNSC based on TP53 mutation status: NT5E expression was more significant in TP53-mutant HNSCC (*P* < 0.05). (e) Promoter methylation level of NT5E in HNSCC: compared with normal tissues, NT5E had a higher degree of methylation in HNSCC (*P* < 0.05). (f) Promoter methylation level of NT5E in HNSC based on TP53 mutation status: NT5E had a higher degree of methylation in TP53 nonmutant HNSCC (*P* < 0.05).

**Figure 3:** (a) Overall survival analysis of NT5E showed that high expression of NT5E significantly reduced overall survival in patients with HNSCC (*P* < 0.05). (b) Disease-free survival analysis of NT5E showed that high expression of NT5E had no significant effect on disease-free survival of HNSCC (*P* = 0.11). (c) The first 25 coexpressed genes of NT5E. (d) The top 25 to 50 coexpressed genes of NT5E. (e) The top 50 to 75 coexpressed genes of NT5E. (f) The top 75 to 100 coexpressed genes of NT5E.

**Figure 4:** (a) GO enrichment analysis of coexpressed genes. In BP, we can see those coexpressed genes were enriched in cell-substrate adhesion, extracellular matrix organisation, extracellular structure organisation, cell junction assembly, and ameboid-type cell migration. Then, in CC, the coexpressed genes were enriched in cell-substrate junction, focal adhesion, and collagen-containing extracellular matrix. At last, in MF, the coexpressed genes were enriched in cadherin-binding, actin-binding, actin filament binding, and so on. (b) KEGG enrichment analysis of coexpressed genes showed that coexpressed genes were mainly concentrated in focal adhesion, PI3K-Akt signalling pathway, regulation of actin cytoskeleton, proteoglycans in cancer, ECM-receptor interaction, MAPK signalling pathway, small cell lung cancer, and bacterial invasion of epithelial cells. (c) Protein-protein interaction network of coexpressed genes. From this network, we can see the interaction in the coexpression mode of CD73. The more lines that connect, the more interactions, which means the gene may be more important. Besides, by using the “CytoHubba” plug-in, we screened out 20 hub genes according to the MCC score.

**Figure 5:** (a) Immune infiltration analysis of NT5E in HNSCC: the expression of NT5E was significantly correlated with B cells, CD8+T cells, CD4^+^ T cells, neutrophils, and dendritic cells in HNSCC. (b) Immune infiltration analysis of NT5E in HPV-positive HNSCC. The expression of NT5E was significantly correlated with B cells, CD8+T cells in HPV-positive HNSCC. (c) Immune infiltration analysis of NT5E in HPV-negative HNSCC. The expression of NT5E was significantly correlated with B cells, CD8^+^ T cells, CD4^+^ T cells, macrophages, neutrophils, and dendritic cells in HPV-negative HNSCC.

**Figure 6:** Validation of NT5E expression in an independent cohort. To further verify the accuracy of our results, we validated the expression of CD73 in an independent cohort. We used the “Ginos Head-Neck” cohort in the Oncomine database to analyse, which is independent for the TCGA cohort. The results showed that CD73 was highly expressed in HNSCC compared with normal tissues (*P* = 5.03E − 7).

## Data Availability

The data that support the findings of this study are available in GEPIA database at http://gepia.cancer-pku.cn and Oncomine database at (http://oncomine.org/).
